# Biochar enhances wheat crop productivity by mitigating the effects of drought: Insights into physiological and antioxidant defense mechanisms

**DOI:** 10.1371/journal.pone.0267819

**Published:** 2022-04-28

**Authors:** Bilal Zulfiqar, Muhammad Aown Sammar Raza, Muhammad Farrukh Saleem, Muhammad Usman Aslam, Rashid Iqbal, Faqeer Muhammad, Jawad Amin, Muhammad Arif Ibrahim, Imran Haider Khan

**Affiliations:** 1 Faculty of Agriculture and Environment, Department of Agronomy, The Islamia University of Bahawalpur, Bahawalpur, Pakistan; 2 Department of Agronomy, University of Agriculture Faisalabad, Faisalabad, Pakistan; 3 National Engineering and Technology Centre for Information Agriculture (NETCIA), College of Agriculture, Nanjing Agriculture University, Nanjing, China; PMAS Arid Agriculture University: University of Arid Agriculture, PAKISTAN

## Abstract

Drought stress is a major limitation in wheat production around the globe. Organic amendments could be the possible option in semi-arid climatic conditions to mitigate the adverse effects of drought at critical growth stages. Wheat straw biochar (BC_0_ = Control, BC_1_ = 3% biochar and BC_2_ = 5% biochar) was used to alleviate the drought stress at tillering (DTS), flowering (DFS), and grain filling (DGFS) stages. Drought stress significantly reduced the growth and yield of wheat at critical growth stages, with DGFS being the most susceptible stage, resulting in significant yield loss. Biochar application substantially reduced the detrimental effects of drought by improving plant height (15.74%), fertile tiller count (17.14%), spike length (16.61%), grains per spike (13.89%), thousand grain weight (10.4%), and biological yield (13.1%) when compared with the control treatment. Furthermore, physiological parameters such as water use efficiency (38.41%), stomatal conductance (42.76%), chlorophyll a (19.3%), chlorophyll b (22.24%), transpiration rate (39.17%), photosynthetic rate (24.86%), electrolyte leakage (-42.5%) hydrogen peroxide (-18.03%) superoxide dismutase (24.66%), catalase (24.11%) and peroxidase (-13.14%) were also improved by biochar application. The use of principal component analysis linked disparate scales of our findings to explain the changes occurred in wheat growth and yield in response to biochar application under drought circumstances. In essence, using biochar at 5% rate could be a successful strategy to promote wheat grain production by reducing the hazardous impacts of drought stress.

## Introduction

Agricultural growth has remained prone to a number of challenges like shrinking arable land, climate change, water shortage, variance in temperature, changes in rainfall pattern, increase in input prices and large scale population shift from rural to urban areas. Therefore, it is need of the time to increase agricultural productivity by the adoption of new tactics in crop production [1,2]. In order to feed the world’s rapidly increasing population, foodstuff production must be doubled by 2050 [3]. Araus *et al*. [4] suggested that rather than expanding the production area in order to increase wheat output, focus on achieving the optimal yield via alternative methods. Constant scarcity of water resources is a significant issue, since it has a severe effect on agricultural production. Additionally, recurrent droughts have impacted more than half of the wheat production area [5,6].

Drought is one of the most detrimental abiotic stress, accounting for the majority of yield losses globally [7]. Wheat is also susceptible to drought stress, particularly during late development stages known as terminal drought. Drought occurs when the atmospheric and soil humidity levels are low and the air temperature is high; this results in a disproportion between evapotranspiration flow and water absorption from the soil [8]. To increase their resistance to oxidative stress, tolerant plants confront a significant challenge in adopting new and improved techniques [9]. There are several factors that influence a plant’s response to drought, including the duration and severity of the stress, the growth stage, the physiological process of growth, and the genotype of the plant [10,11], environmental factors [12,13], photosynthesis mechanism activation [14,15], and various patterns of gene expression and respiration activity [16].

Global warming and its associated climatic consequences have a detrimental influence on the globe. Biochar use and production are critical in agriculture for reducing climate change and improving the quality and management of agricultural and forestry waste. Alburquerque *et al*. [17] defined biochar as a carbon-containing substance obtained via the pyrolysis of biomass residues. Additionally, Ahmad *et al*. [18] concluded that biochar is a viable option for resolving drought-related problems.

Lehmann and Joseph [19] claimed that biochar has the potential to significantly improve and remediate soil and water functions such as adsorption capacity, CEC, organic carbon content, water holding capacity, mechanical strength, and nutrient retention ability. In summary, biochar is said to improve the fertility, quality, and enzyme activity of soil. Additionally, owing to the specific properties of biochar, it is critical for the elimination of aquatic pollutants, toxins, and steroids [20].

Biochar (BC) is generated by pyrolyzing organic matter in a low-oxygen environment and is garnering significant attention as a soil supplement globally because to its potential to bind heavy metals, act as a carbon sink, and decrease greenhouse emissions to help combat climate change [21,22]. Numerous examples exist in the literature describing the beneficial effects of BC in the presence of trace elements [23,24]. Additionally, BC has been shown to improve soil water retention capacity but not available soil water content [25]. Biochar improved maize production, soil base saturation, and the amount of water accessible to plants [26].

The soil application of BC has been reported to improve the growth and yield of sunflower [27], rapeseed [28] and wheat [29] under drought stress conditions. Biochar enrichment significantly improved the stomatal conductance, water use efficiency and photosynthesis in tomato crop under water scarce conditions [30]. Furthermore, an increase in osmotic potential, photosynthetic rate, transpiration rate, relative water contents, leaf water potential and leaf turgor potential under drought conditions has been reported by Haider *et al*. [31] and Haider *et al*. [29] and Kammann *et al*. [32] in maize, wheat and quinoa, respectively. It has been publicised that BC application mitigates the negative effects of drought by improving the electron transfer and protective enzymes activity in crops Lyu *et al*. [33].

Biochar is the most feasible alternative to cope up drought conditions for sustainable agriculture production due to its long-term carbon sink in the soil, high porosity, cation exchange capacity and ability to serve as a home for beneficial microbes [14,26,27]. Its soil application improves the water and nutrient holding capacity of soil, seed germination, seedling emergence, productivity, microbial activity, and other chemical processes in soil [34–36]. Therefore, the application of biochar could be a step forward in ameliorating the adverse effects of drought on critical growth stages of wheat.

We hypothesize that biochar soil application will improve soil characteristics, growth, water-related parameters, physiological attributes and productivity of wheat under drought conditions.

## Materials and methods

### Experimental layout and crop husbandry

The experiment was conducted in The Islamia University of Bahawalpur, Pakistan (Latitude: 29° 23’ 60.00” N, Longitude: 71° 40’ 59.99” E) and was replicated four times using a randomised complete block design (RCBD) under factorial setting. Three biochar treatments were applied at each studied growth stage as following: BC_0_ (control), BC_1_ (3% w/w biochar, 180 g pot^-1^), and BC_2_ (5% w/w biochar, 300 g pot^-1^) [37]. Drought was imposed at tillering (DTS), flowering (DFS), and grain filling (DGFS) stages, while full irrigation was considered as control.

Wheat seeds (Galaxy 2013) were obtained from the Regional Agricultural Research Institute (RARI) Bahawalpur, and planted in plastic pots (26×29 cm) filled with 6 kg sieved biochar mixed soil on November 9th, 2019. The physiochemical analysis of soil is given in Table 1. A clear plastic sheet was placed over the wire house to protect the plants from rain, when required. All pots were evenly watered until full emergence. Four plants per pot were maintained by uprooting extra plants after 20 days of sowing.

**Table 1:** Physical and chemical properties of the experimental soil.

Parameters	Soil Profile
Sand	61%
Silt	33.5%
Clay	11%
Texture class	Sandy loam soil
Ph	7.23
Electric conductivity (dSm^-1^)	2.55
Ammoniac N (mg g^-1^)	1.58
Organic matter (%)	0.92
Available Phosphorus (ppm)	6.75
Available Potassium (ppm)	112

### Biochar application and drought imposition

The biochar was produced by pyrolyzing wheat straw at 500°C in a vertical kiln as described by [38], having following properties: particle size 3 mm, bulk density 0.53 g cm^-3^, micropore surface area 73.6 m^2^ g^-1^, micropore volume 0.024 cc g^-1^, cation exchange capacity is 13.4–14.8 c mol kg^-1^, ash content 20.7% and pH 9.1 [29].

Every pot was watered in the same way since the drought began. Following that, 30% pot water holding capacity (WHC) was maintained under drought at tillering (DTS), flowering (DFS), and grain filling (DGFS) stages, whereas 80% pot WHC was considered as a control.

### Recorded parameters

#### Growth and yield parameters

Growth and yield related parameters such as plant height (cm), spike length (cm), number of grains per spike, 1000-grain weight (g), biological yield per plant (g), and grain yield per plant (g) were recorded as per standard procedures/protocols. The harvest index (HI) was calculated as per following formula:

$$HI=\frac{Grain\;Yield}{Bilogical\;Yield}\times 100$$

#### Determination of physiological parameters

Hashem and El-Sherif [39] extracted the photosynthetic pigments chlorophyll (Chl a) and chlorophyll (Chl b) in 80% (v/v) acetone and quantified them spectrophotometrically. A portable pulse amplitude modulation fluorometer was used to determine the fluorescence of chlorophyll in leaves (Handy PEA. Hansatech. Norfolk, UK). The leaves were dark adapted in a leaf clip for 30 minutes. Thirty measurements were collected for each treatment (three replicates of 10 leaves from different plants). The water use efficiency (WUE) was calculated by the formula described by Raza *et al*. [36] WUE = grain yield/total water applied. Stomatal conductance (SC) was measured by using an automatic porometer MK-3 Delta-T Devices, Burwell Cambridge, England.

#### Determination of electrolyte leakage and hydrogen peroxide concentration

Oxidative stress and antioxidant enzyme activity were determined 65 days after planting. Electrolyte leakage % (EL) in shoots was measured by putting samples vertically in tubes and heating in a known amount of distilled water at a constant temperature of 32°C for 2 hours, after which the EC solution was calculated as EC1 and the solution was heated at another constant temperature (121°C) for 20 minutes, after which the EC solution was estimated as EC2. Finally, the EL was computed using an equation that had previously been established [40].


$$EL=\frac{EC1}{EC2}\times 100$$

For hydrogen peroxide (H_2_O_2_) measurement, 3.0 mL of phosphate buffer solution was added to a 50 mg sample and centrifuged for 30 minutes at 4°C and 6000 g. Following that, the supernatant was added to 1.0 mL of titanium sulphate (0.1%) and centrifuged at 6000 g for 20 minutes at 4°C. At 410 nm, the supernatant’s absorbance was determined. H_2_O_2_ was calculated using an extinction coefficient of 0.28 mol^-1^ cm^-1^.

#### Estimation of antioxidant enzymes

The superoxide dismutase (SOD) activity was determined according to the method described by Giannopolitis and Ries [41]. To a 3 mL reaction mixture containing 50 mM phosphate buffer (pH 7.8), 13 mM methionine, 75 μM nitro blue tetrazolium, 0.1 μM EDTA, and 0–100 μl of enzyme extract was added 2 μM riboflavin. The tubes were shaked and illuminated with a 15-W fluorescent tube. The reaction was allowed to run for 10 min after which the light was switched off and the absorbance read at 560 nm. One unit of SOD activity was defined as the amount of enzyme required to cause 50% inhibition of the rate nitroblue tetrazolium chloride reduction.

Hwang *et al*. [42] proposed a technique for estimating CAT activity by measuring the rate of decomposition of H_2_O_2_ at 240 nm. POD activity was measured according to the guaiacol oxidation method described by Maehly and Chance [43] with small modification: 3 ml reaction mixture consisted of 50 mM potassium phosphate buffer (pH 6.1), 1% guaiacol, 0.4% H_2_O_2_ and enzyme extract. Increase in the absorbance due to oxidation of guaiacol (E = 25.5 mM^–1^ cm^–1^) was measured at 470 nm [44].

#### Statistical analysis

STATISTIX software (version 8.1) was used on the current data to determine the analysis of variance (ANOVA), and the least significant difference (LSD) at 5% probability level was used for mean data comparison [45]. The data were subjected to principal component analysis (PCA) and biplot graph was developed through Origin Pro 9.1 software to examine the results of this analysis.

## Results

### Plant height and spike length

Drought stress significantly reduced plant height by 52, 42.9, and 28% and spike length by 40%, 38%, and 30% at tillering, flowering, and grain filling stages, respectively, when compared with control treatment. Application of biochar (BC_1_ and BC_2_) alleviated the drought stress and increased plant height and spike length by 9, 15.7, and 11.9, 16.6%, respectively (Table 2).

**Table 2:** The effect of biochar on plant height (PH, cm), spike length (SL, cm), number of grains per spike (NGPS), 1000-grain weight (GW, g), grain yield (GY, g pot^-1^), biological yield (BY, g pot^-1^), harvest index (HI) of wheat under drought stress.

Treatments	BC Application	PH	SL	NGPS	GW	GY	BY
**CK**	**BC**_**0**_	60.66 b	9.94 b	33.67 bc	30.67 c	6.93 a	15.20 b
	**BC**_**1**_	63.66 ab	11.07 a	35.67 b	33.00 b	7.23 a	15.82 ab
	**BC**_**2**_	66.67 a	11.56 a	38.67 a	35.33 a	7.56 a	16.26 a
**DTS**	**BC**_**0**_	38.00 h	7.10 h	27.67 ef	25.50 fg	5.36 cde	11.50 def
	**BC**_**1**_	41.33 g	7.76 fg	30.33 d	27.67 de	5.70 bcd	12.25 cde
	**BC**_**2**_	46.00 ef	8.33 de	33.00 c	29.00 d	6.13 b	12,77 c
**DFS**	**BC**_**0**_	32.33 i	6.96 h	28.00 ef	24.67 g	5.46 bcde	11.40 ef
	**BC**_**1**_	44.33 fg	8.03 ef	30.33 d	26.33 ef	5.73 bcd	12.17 cde
	**BC**_**2**_	49.00 df	8.53 cde	33.33 c	27.56 de	5.93 bc	12.44 cd
**DGFS**	**BC**_**0**_	36.67 h	7.23 gh	26.33 f	23.00 h	4.96 e	10.50 f
	**BC**_**1**_	51.00 d	8.67 cd	27.67 ef	25.00 fg	5.23 de	11.08 f
	**BC**_**2**_	54.67 c	9.03 c	29.33 de	26.33 ef	5.90 bcd	12.50 cd
**LSD (p < 0.05)**		**3.07**	**0.56**	**2.24**	**1.57**	**0.67**	**1.02**

CK, DTS, DFS and DGFS indicates control, drought at tillering, flowering and grain filling stages respectively. BC_0_, BC_1_ and BC_2_ indicates control, 3% and 5% biochar respectively. Means sharing the same letter case are not significantly different at 5% probability level.

### Yield attributes

Drought stress at critical growth stages (DTS, DFS, and DGFS) reduced the number of spikelets per spike (28.3, 31.1, and 40.6%), the number of fertile tillers (21.5, 25.8, and 32.3%), the number of grains per spike (18.6, 17.8, and 29.6%), the 1000 grain weight, the grain yield (29.3, 31.5, and 40.6%), the biological yield (10.2, 18.4, and 23.7%), and the harvest index. Biochar had a beneficial impact in either drought or control circumstances, reducing drought effects or raising the values of the aforementioned parameters. However, BC (5%) application results in a greater grain yield (10.4%) than BC 3% application. Biochar treatment substantially decreased the impact of drought on yield-related characteristics of wheat such as spikelet count per spike, fertile tiller count per spike, grain count per spike, 1000 grain weight, grain yield, biological yield, and harvest index (Table 2).

### Water use efficiency and stomatal conductance

Water shortage increased the efficiency of wheat water consumption when biochar was applied at different development stages, as indicated in Fig 1. WUE dropped by 42, 45, and 34% under drought stress at DTS, DFS, and DGFS, respectively, compared to the control treatment. Biochar (BC_1_ and BC_2_) significantly reduced the drought impact by 25% and 38%, respectively, as compared to no biochar treatment. Similarly, stomatal conductance (m mol m^-2^ s^-1^) dropped by 10.5, 20.7, and 27.2% under drought stress at DTS, DFS, and DGFS, respectively, compared to the control treatment. Moreover, BC_1_ and BC_2_ significantly reduced the drought impact by 28.7% and 42.8%, respectively, as compared to the control treatment.

**Fig 1:** Water use efficiency (%) and stomatal conductance (m mol^-2^ s^-1^) contents affected by biochar application under drought stress at critical growth stages of wheat. CK, DTS, DFS and DGFS indicates control, drought at tillering, flowering and grain filling stages respectively. BC_0_, BC_1_ and BC_2_ indicates control, 3% and 5% biochar respectively. Error bars indicates standard error (n = 4).

### Chlorophyll concentrations

Biochar treatment had a substantial effect on the chlorophyll content (a and b) of wheat leaves subjected to drought stress (Fig 2). When compared to the control treatment, the addition of biochar (3 and 5%) raised the chlorophyll contents a and b by 13, 19% and 11.2, 22.1%, respectively. While drought stress diminished Chlorophyll a and b by 34.8, 31.8, 21.0% and 36.6, 39.2, 42.7%, respectively, when compared to no biochar treatment at critical growth stages (DTS, DFS and DGFS) of wheat. Under stressful circumstances, 5% biochar application resulted in more substantial effects.

**Fig 2:** Chlorophyll a and b (mg g^-1^ FW) contents affected by biochar application under drought stress at critical growth stages of wheat. CK, DTS, DFS and DGFS indicates control, drought at tillering, flowering and grain filling stages respectively. BC_0_, BC_1_ and BC_2_ indicates control, 3% and 5% biochar respectively. Error bars indicates standard error (n = 4).

### Gas exchange attributes

Transpiration and photosynthesis rate were significantly dropped by 74.5, 69.5, 62.8 and 43.5, 32.4, 31.1% under drought stress at DTS, DFS, and DGFS, respectively, as compared to the control treatment. Moreover, stomatal conductance decreased positively under water stress by 10.5, 20.7 and 27.2% at DTS, DFS, and DGFS. Biochar treatment had a substantial effect on the gas exchange attributes of wheat leaves subjected to drought stress (Fig 3). BC_1_ and BC_2_ significantly enhanced the transpiration and photosynthesis rate by 27.8, 39.1% and 17.6, 24.8%, respectively when compared with control. Similarly, BC_1_ and BC_2_ significantly improved stomatal conductance by 28.6 and 42.7% as compared to control. BC_2_ application performed best result than other treatments under drought.

**Fig 3:** Photosynthetic rate (μmol CO_2_ m^-2^S^-1^) and transpiration rate (mmol H_2_O m^-2^S^-1^) affected by biochar application under drought stress at critical growth stages of wheat. CK, DTS, DFS and DGFS indicates control, drought at tillering, flowering and grain filling stages respectively. BC_0_, BC_1_ and BC_2_ indicates control, 3% and 5% biochar respectively. Error bars indicates standard error (n = 4).

### Oxidative stress and antioxidants

Under drought stress, the higher amount of EL and H_2_O_2_, 19.8, 13.9, 11.0% and 17.6, 22.4, and 29.8%, were found during the DTS, DFS, and DGFS stages of wheat respectively. BC treatment substantially decreased the levels of EL and H_2_O_2_ in the leaves. In drought circumstances, a 5% application of biochar outperformed a 3% treatment by a considerable margin Fig 4.

**Fig 4:** Hydrogen peroxide (μM g^-1^ FW) and Electrolyte leakage (%) affected by biochar application under drought stress at critical growth stages of wheat. CK, DTS, DFS and DGFS indicates control, drought at tillering, flowering and grain filling stages respectively. BC_0_, BC_1_ and BC_2_ indicates control, 3% and 5% biochar respectively. Error bars indicates standard error (n = 4).

The application of biochar during drought also had a substantial effect on the antioxidant activities of wheat leaves as shown in Figs 5 and 6. Drought enhanced CAT and SOD activity while reducing POD activity, but substantially boosted biochar use during the DTS, DFS, and DGFS phases. CAT and SOD activity were decreased by 19.1, 11.6, 14.7, and 21.2, 16.2, and 28.9%, respectively, while POD levels were decreased by 5.9, 4.2, and 2.1%, respectively. Furthermore, BC_2_ (5%) application was more effective than BC_1_ both under drought and control treatments.

**Fig 5:** Catalase (μmol min^-1^ mg^-1^ protein) and Superoxide dismutase (μmol min^-1^ mg^-1^ protein) activities affected by biochar application under drought stress at critical growth stages of wheat. CK, DTS, DFS and DGFS indicates control, drought at tillering, flowering and grain filling stages respectively. BC_0_, BC_1_ and BC_2_ indicates control, 3% and 5% biochar respectively. Error bars indicates standard error (n = 4).

**Fig 6:** Peroxidase (μmol min^-1^ mg^-1^ protein) activities affected by biochar application under drought stress at critical growth stages of wheat. CK, DTS, DFS and DGFS indicates control, drought at tillering, flowering and grain filling stages respectively. BC_0_, BC_1_ and BC_2_ indicates control, 3% and 5% biochar respectively. Error bars indicates standard error (n = 4).

### Principal component analysis

Principal component analysis (PCA) was performed on all the studied traits in order to discover their correlations with the most relevant treatments and other variables. In terms of wheat grain yield and its contributing traits, there was no clear separation between PC_1_, which accounted for 93.49% of the variation, and PC_2_, which was found in PCA. PC_1_ (84.36%) and PC_2_ (9.13%) accounted for the majority of the variance in the loading and score plots. As depicted in Fig 7 obtuse and acute angles indicate a negative or positive association between two trait vectors, respectively, while a right angle between two variable vectors indicates no correlation at all. Cosine angle According to a biplot graph created using PCA analysis, GY and its contributing attributes were found to have a strong correlation with antioxidants and gasses exchange attributes (SOD, POD, CAT, WUE, EL%, H_2_O_2_).

**Fig 7:** Plotting a PCA biplot shows 93.49% of the data’s variability. For example, the cosine angle indicates correlation between traits; acute and obtuse angles indicate positive and negative associations; while a right angle between two vectors of variables indicates no correlation. An example of a biplot is shown below. It shows the relationships between various parameters such as grain yield (GY) and biological yield (BY), as well as other factors such as plant height (PH) and the number of fertile tillers (NFT), shoot length (SL) and the number of spikelets per spike (NSPS) and number of grains per spike (NGPS), 1000 grain weight (1000GW), transpiration rate (Tr), photosynthetic rate (Pr), water use efficiency (WUE), Chl a (Chlorophyll a), Chl b (Chlorophyll b), EL% (Electrolyte leakage %), H_2_O_2_ (Hydrogen Peroxide), CAT (Catalase), POD (Peroxidase), SOD (Superoxide Dismutase) of wheat crop under drought at tillering (DTS), flowering (DFS), and grain filling stages (DGFS) and full irrigation as control (CK) by using three biochar treatments such as BC_0_ = control, BC_1_ = 3%, and BC_2_ = 5%.

## Discussion

Plant height was considerably reduced under drought stress at critical growth stages of wheat. Similar findings have been reported by Raza *et al*. [46] and Zhao *et al*. [47] in wheat and *Brassica napus* under water-stress, respectively, which is in consistent with our findings. Plant cell dehydration and reduced turgidity cause altered protoplasmic activities, which reduce cell division and result in lower plant height [48,49]. When compared to the control, the higher application of BC during a drought dramatically boosted plant height of wheat. The application of a greater dose of biochar (5%) resulted in a significant increase in plant height. Haider *et al*. [29] found similar findings concerning the favourable impacts of biochar on plant height in wheat crop, as it promotes nutrient absorption, soil microbial activity, photosynthetic rate, and hence plant height [36,50].

Wheat straw biochar has a positive influence on crop growth and production. Several growth and yield parameters like shoot length, spike length, grain yield, biological yield, and harvest index of wheat were reduced under drought conditions. The application of biochar mitigated the adverse effects of drought on the above mentioned attributes. The findings of Haider *et al*., [29] are also in line with our results that biochar application improved the growth and yield of wheat both under control and drought conditions. BC treatment improved soil structure, which benefited plant growth and development [26]. Iqbal *et al*. [51] reported that water-stress reduced spike length by lowering plant metabolic activity [52]. The use of biochar boosted the nutritional availability and source sink relationship which in turn increased spike length and ultimately grain yield [53]. Biochar application improves the water, carbon and reduce Na^+^ uptake from soil that improves metabolic functions, biomass production, and yield of wheat [35].

The present study illustrated that water scarcity reduced photosynthetic activity and stomatal conductance, leading in decreased moisture content under drought stress. The addition of biochar to soil boosted cation exchange capacity as well as physicochemical qualities hence increased photosynthetic rate and accessible soil water which are in accordance with Khan *et al*. [54] and Hafez *et al*. [55]. Leaf chlorophyll content, gas-exchange characteristics, WUE, SC and transpiration rate were decreased under drought stress than well watered plants. Similar findings have been reported by Zaheer *et al*. [56] and Raza *et al*. [57] in wheat crop due to partial stomatal closure. Biochar mitigated drought impacts by keeping water in the pores and gently releasing it under dry conditions [25]. Notably, the pH of the soil was altered by the application of biochar which nutrient absorption and availability in rhizosphere [58].

Drought stress in wheat increased the EL, H_2_O_2_ concentration and POD activity whereas reduced the SOD and CAT activity. SOD has been found to convert O_2_ to H_2_O_2_ directly and CAT to H_2_O_2_ and O_2_ directly, and POD may play a significant part in H_2_O_2_ catalysis. Reactive oxygen species (ROS) detoxification is feasible in plants and a balance of ROS generation and breakdown is required for optimal plant development [59,60]. However, plants are unable to detoxify ROS, especially under stressful conditions, leading to oxidative stress in plants [21]. Lipid peroxidation and nucleic acid damage are two of the major ways in which oxidative stress may interfere with a plant’s biological activity [59,61]. Multiple plant species were shown to suffer from oxidative stress due to water scarcity [7]. Biochar amendments improved the SOD, POD and CAT activities by improving plant metabolic functions, cell growth, reducing ROS production and better soil plant and water relations [62–64]. Biochar has the capability to enhance cation exchange capacity, physiochemical properties and soil water and nutrient holding capacity and hence improve the growth and yield of crops [65,66].

## Conclusion

Drought stress significantly reduced the growth and yield of wheat crop. Soil biochar application mitigated the harmful effects of drought by improving soil fertility, water and nutrient holding capacity of soil and source sink relationship in crops. BC application improved the growth, physiological, water related parameters and yield of wheat both under control and drought conditions. Furthermore, grain filling stage was found more sensitive to drought and biochar soil application is the best option to cope up the negative effects of drought in wheat.
